The article "A Recommendation Model for College English Digital Teaching Resources Using Collaborative Filtering and Few-Shot Learning Technology" was published in 2022. Journal: Comput Intell Neurosci.

# A Recommendation Model for College English Digital Teaching Resources Using Collaborative Filtering and Few-Shot Learning Technology

**DOI:** 10.1155/2022/1233057

**Published:** 2022-07-01

**Authors:** Juan Li

**Affiliations:** Baotou Medical College, Inner Mongolia University of Science and Technology, Baotou 014040, China

## Abstract

This study designs and implements a digital English instructional resource management recommendation system based on collaborative filtering technology based on CF research and the construction of digital English instructional resources. This study designs the system with *B*/*S* structure combined with hierarchical design architecture, plans the overall design goal, architecture design, compilation structure, and key technologies, and designs and implements the system's core modules on the basis of fully analysing the functional and nonfunctional requirements of personalized educational resource recommendation system. Furthermore, the traditional CF has been improved to address scalability, data sparseness, and user cold start in the recommendation process. The evaluation results show that this algorithm has a recall rate of 96.37% and a system resource recommendation accuracy rate of 95.31%, both of which are higher than the traditional method's 6.37%. This algorithm can overcome the drawbacks of traditional algorithms, improve recommendation accuracy, and efficiently provide high-quality English teaching resources. Educators and students will be more likely to find high-quality digital English instructional resources if they use the instructional resource system proposed in this study.

## 1. Introduction

The use and development of digital technology have ushered in a technological revolution in the world of education. It has an impact on education, resulting in significant changes in educational and learning methods [1]. The result of the digitalization of teaching media is digital instructional resources. In the field of online education, particularly in the teaching environment, digital instructional resources have become indispensable. The information, digitalization, and networking era have posed a challenge to traditional college English instruction. The need for college English teaching reform is critical in order to adapt to the new situation and requirements [2]. The goal of digitalizing English knowledge is to divide it into manageable chunks, allowing students to customise, acquire, and organise the platform as they see fit. It is an English decomposition and matrix assembly process that assists students in establishing English logic and thinking as well as internalising English into habits by effectively connecting and bearing various knowledge such as society, life, major, and workplace [3]. People gradually realize that digital and multimedia network technology can be organically integrated with education and teaching. Digital technology provides technical support for delivering a variety of required scenarios that can vividly show phenomena and processes that are difficult to express in traditional teaching modes, as well as vividly express abstract content and guide learners to intuitively feel abstract language concepts [4]. In today's Internet age, the degree of educational informatization, the digitization of instructional resources, and the efficacy of their application have gradually become an important symbol for evaluating a country's or region's educational modernization process. With the advent of the Education 4.0 era, the creation and use of digital resources in English teaching will become more common [5]. Building and perfecting a digital college English instructional resource database can help college English teachers better accomplish their goals and develop English professionals who are well rounded in listening, speaking, reading, writing, and translation.

The acquisition range of college English instructional resources has greatly expanded in the information environment. It can now be extended to all of the world's instructional resources, not just those in schools and China. The abundance of instructional resources also encourages teaching mode innovation. The term “instructional resource bank” refers to a resource bank that can meet teaching requirements, has rich and diverse teaching content that adheres to specific requirements and norms, and is convenient for professors to impart knowledge and recipients to learn more effectively [6]. Digitalization of instructional resources in the information environment is easier to integrate than books, newspapers, and other written materials, which is beneficial to the role of resource allocation. Driven by reform power and teaching demand, all universities have set up their own instructional resource banks and network electronic resources to varying degrees after practice and development [7]. However, nowadays, the creation of digital resources frequently follows a centralised and unified management model, in which each university creates its own resource bank. As a result, each digital instructional resource bank and resource management system are relatively self-contained, and their resources are essentially closed off from one another, resulting in information barriers and islands [8]. The current research focus is on how to solve the problem of information isolation and personalized resource recommendation. Personalized recommendation services are now widely used in a variety of industries. Collaborative filtering technology is currently the most studied and widely used recommendation system, as well as a personalized recommendation system with high recommendation efficiency. Many mixed recommendation methods use collaborative filtering technology, according to research and analysis of the current personalized recommendation literature. In the recommendation process, CF (collaborative filtering) algorithm does not need to extract the content features of items and can make cross-domain recommendations, resulting in a high level of personalization and automation. This study focuses on the creation and implementation of CF-based digital English instructional resources. The following are some of its innovations:

① Based on the project characteristics of digital English instructional resources, this study designs a specific instructional resource recommendation process. When searching for the nearest neighbor of the target user, considering the relationship among users, resources, and resource attributes, the method of combining the similarity of rating with the similarity of preference of resource attributes is adopted, making full use of effective information to mine out more similar users, improving the recommendation quality of the system and solving the problem of data sparsity.
② According to the principle, advantages, and disadvantages of collaborative filtering recommendation algorithm in personalized recommendation technology, combined with learners' learning behavior characteristics, this study constructs a digital English instructional resource management recommendation model. In the construction of user model, the system extracts the features of users' personalized resource access to form an individual user model and clusters users with similar interests to form a group user model. Finally, an integrated user interest vector is formed to construct an integrated user model. This system provides a good solution for a personalized recommendation of digital English instructional resources.

This study is divided into five sections based on the research requirements: the first section is the introduction. This section explains the research's content, significance, methods, and definitions of related concepts and provides a quick overview of the study's structure. The second section is the literature review. This section summarises relevant literature from both domestic and international sources, as well as the study's research ideas and methods. The third section is methodology. This section explains the concept, types, and characteristics of English educational resources; this study examines the current state of English educational resource construction; a recommendation system for managing English instructional resources based on CF is developed, along with the implementation process. The fourth section conducts an experiment with the model developed in this study, analysing its performance and practical application impact. The fifth section is a summary and outlook. This section begins by summarising the research work of this study, explaining the findings, and then looking ahead to future research work and prospects.

## 2. Related Work

Network teaching relies heavily on the creation of digital instructional resources. Each website has formed a certain scale of instructional resources as a result of the establishment of various websites of instructional resources. However, how to find interesting information from a large number of instructional resources quickly and effectively remains a problem. Personalized recommendation services have a bright future in the information age, and they offer a fresh perspective on the instructional resource system. More platforms are introducing recommendation systems to provide personalized services to users, and many scholars and experts have devoted themselves to recommendation system research, with excellent results.

Li designed a flexible, reliable, high-performance personalized recommendation system architecture that can store and process petabytes of data and make real-time recommendations [9]. Osipov et al. proposed an intelligent online learning recommender system that can self-evolve while achieving self-adaptation to learners and an open network environment [10]. The information resources existing in the system are not fixed, and the learning resources on the network can be integrated into the system according to the interaction between users and the system. Kambanaros et al. analysed the user's browsing behavior and preference information by sampling and then presented the generated instructional resource recommendation list to the user, effectively realizing the sharing and recommendation of resources [11]. Davis studied the application of collaborative filtering technology in the personalized recommendation system of scientific literature and proposed two methods of collaborative recommendation [12]. One is a collaborative recommendation algorithm based on ontology concepts and user interests, and the other is a collaborative recommendation algorithm based on weighted association rules. Hafner pointed out that the existing network instructional resource system has not really applied the personalized recommendation technology and is only in the research stage. With the continuous enrichment of instructional resources, the need to realize personalized recommendation service of network instructional resource system is more and more urgent [13]. Shi and Yang proposed a method for real-time recommendation of current and subsequent learning materials based on learner interests and progress [14]. The method is implemented through three links: data and processing, mining neighbor learners, and recommendation of learning materials. Gee et al. proposed an online automatic recommendation system based on a hybrid filtering recommendation technique. The system combines content-based filtering and collaborative filtering to make recommendations based on the user's recent navigation history [15]. Yuan builds a user interest model by combining explicit tracking and implicit tracking of users [16]. Nielsen and Hoban applied web mining, association rule mining, and decision tree techniques to recommender systems to recommend suitable resources to users [17]. Arnaiz-González et al. studied the personalized resource recommendation service in the basic education resource network and proposed a personalized resource recommendation service model [18]. Aiming at the contradiction between the current ubiquitous mass instructional resources and the personalized needs of users, Barry proposed to introduce personalized recommendation technology into the network instructional resource system [19]. The system fully pays attention to the individual differences of learners and provides users with personalized services according to the learners' learning background and interests. For the sparsity problem of rating data, Cazden proposed that the dimensionality of item space can be reduced by using the singular value decomposition technique, thereby improving the sparsity of user rating data [20].

This study examines CF and related literature in the field of instructional resource construction, as well as personalized recommendation technology. A recommendation system for English instructional resource management based on CF is designed based on the foregoing. The algorithm chooses the user with the greatest distance as the initial clustering centre, divides users with similar resource attribute preferences into the same cluster through offline clustering, and searches the nearest neighbors in several clusters close to the target user, reducing the time and space cost of neighbor query. The flexible data processing ability of Spark and Hadoop technologies is realized in this study, and the discipline classification tree is constructed to form a better organisational resource model and user model of tagged data sources. The cold start problem is solved and the algorithm's accuracy is improved by using a hybrid recommendation algorithm based on content and collaborative filtering. The experiment demonstrates that the research presented in this study can aid in the creation and sharing of digital instructional resource databases and improve learners' learning efficiency.

## 3. Methodology

### 3.1. Digital English Instructional Resources

Digital instructional resources refer to all kinds of materials or systems that are processed digitally, support the effective operation of teaching, realize the teaching purpose, and can run on the computer or network environment [21]. It can reduce the macroworld, enlarge the microworld, turn the abstract into the concrete, turn the virtual into reality, and put history, future, and present into operation at the same time. It can fully arouse students' positive thinking in all senses. It can enable students to find and share digital knowledge and information resources through independent or creative ways, realize multilevel communication, evaluation, and exchange, and stimulate students' interest in learning. The design of digital instructional resources has two contents, one is the organisational design of instructional resources and the other is the description information design of instructional resources. In order to make the best use of digital English instructional resources, digital English instructional resources must be designed concisely, easy to understand, and operate. Some fashion elements can be added to the resource library to attract students. At the same time, it is necessary to fully consider the description of the resources themselves, that is, the design of descriptive information of instructional resources. Generally, it should include overall description, history and current situation description, metadata description, teaching characteristics description, ownership description, generic information description, and quality information description [22]. The particularity of digital English instructional resources lies in the following aspects: ① dealing with digitalization and realizing the quantification and standardization of information. ② Network transmission, clear information support points and links, and establishing an information chain. ③ Intelligent retrieval to meet the demand of customised information acquisition. ④ Multimedia presentation and realizing multilayer simultaneous stimulation such as audiovisual and speaking. ⑤ Hyperlinking of organisation, which realizes platform-type hyperlink of various information and resources and completes the knowledge structure. The digital college English instructional resource management model is shown in Figure 1.

The depth and breadth of college English textbooks and courseware are currently lacking [23]. Many teachers discover that the format of courseware solidifies over time. As a result, the digital English instructional resource database must use the existing or under-construction campus network to provide teachers with access to instructional resources and to aid in the teaching of students' English listening, speaking, reading, writing, and translation skills. Multimedia materials, teaching software, a network platform, and an integrated teaching system are just a few of the digital English instructional resources available. These digital resources can be organised by classifying knowledge points, teaching emphasis or difficulty, or knowledge and skill. It is important to note that the goal of digitalizing English knowledge is to divide it into manageable chunks so that students can customise, acquire, and organise the platform as they see fit. It is an English matrix assembly and linear decomposition process. It can assist students in developing English logic and thinking, as well as internalising English into habits, by effectively connecting and bearing various types of knowledge, such as society, life, major, and workplace. Learning resources in the network differ from traditional books and teaching materials due to the digitalization of learning objects. Traditional instructional resources are blocked and rigid due to the lack of digital media technology, making information sharing and transmission difficult. Learning objects that have been digitalized can help with the effective transmission of learning materials and resource sharing [24]. Digital instructional resources provide vivid and intuitive learning materials for students; through a large number of repeated information input, listening and speaking training becomes easy, thereby arousing the enthusiasm of students' classroom participation and promoting classroom interaction. It overcomes the passive situation of students in traditional classroom teaching and provides an effective guarantee for improving students' listening and speaking abilities. In the functional application of digital English instructional resources, teachers and students are more dependent on retrieval function and interactive function.

### 3.2. CF

This section mainly introduces the recommendation system and common collaborative filtering recommendation technology in detail. In the traditional system platform, the user browsing platform can only passively receive the information provided by the platform. Because of the different needs of each user, it cannot serve every user. With the development of educational informatization, the number of instructional resources on the Internet is also increasing [25]. Information technology has become increasingly difficult to help users find the resources they need. The personalized recommendation technology changes the system from a passive information provider to providing users with interesting information, which is more targeted than the traditional way. A personalized recommendation system can free users from massive information and greatly save the time and cost of finding commodities. At present, personalized service has become a new research hotspot in intelligent information processing and network technology. Personalized recommendation technology can analyse and predict users' behavior by collecting and analysing users' information, so as to better provide users with their corresponding services and achieve the purpose of personalized service. From the overall hierarchical structure, the recommendation system is mainly composed of three modules: ① *Input Function Module*. Its main function is to collect and update data and do some preprocessing work to improve data quality. ② *Recommendation Algorithm Module*. It is the core and part of the recommendation system, through which users will get the final recommendation result. ③ *Output Function Module*. The results obtained by the recommendation algorithm module are displayed to users through this module.

The personalized recommendation algorithm is at the heart of the system, and it plays a critical role in recommendation quality. When selecting a personalized recommendation algorithm, it is necessary to weigh the benefits and drawbacks of various recommendation algorithms in light of the application field's unique characteristics in order to select the most appropriate recommendation algorithm for this application. A good recommendation algorithm can improve the performance of a recommendation service, find the information users require quickly and accurately, and increase resource utilisation and website service quality. User statistics-based recommendation, content-based recommendation, and collaborative filtering recommendation are the three types of personalized recommendation technology currently available. Users should be able to express their needs easily, and personalized recommendation systems should actively recommend resources to them. The system can adapt to changing user requirements over time. The advantage of a recommendation based on user statistics is that it does not rely on user behavior information, so there is no cold start problem. It can be used internally in a variety of fields because it is not dependent on the resource's information. In the field of information retrieval, content-based recommendation is proposed. Content-based recommendation is a recommendation method that was previously used with personalized recommendation technology. Content-based recommendations are based on the assumption that items that are similar in content to information items that the user was interested in previously will remain interesting to the user in the future. The basic idea behind content-based recommendation is to assess users' behaviors and needs based on the content they have access to. User interest files are used to describe each user's interests; a feature vector is created by extracting the features of each resource's information content; the recommendation system recommends resources based on similarity. This recommendation mechanism is more accurate than the statistical recommendation method of users because it can model the user's preference resources well.

The principle of collaborative filtering recommendation is to find the correlation between resources or between users according to their preferences for items or resources and then make recommendations based on these correlations. Collaborative filtering recommendation is mainly divided into user-based recommendation and project-based recommendation. The basic idea of collaborative filtering is very intuitive. In daily life, people often make some choices such as shopping, reading, and music according to the recommendations of friends and relatives. Collaborative filtering technology is to apply this idea to information recommendation and recommend a certain user based on other users' evaluation of certain information. Generally speaking, collaborative filtering needs to solve two problems: ① how to determine the user groups with similar interests and ② how to predict the resources or items that users are interested in. There are three basic starting points: ① users can be classified according to their interests, ② the user's rating information on the project includes the user's interest information, and ③ users' ratings of unevaluated items are similar to those of similar users. The structure of English instructional resource management recommendation system based on improved CF is shown in Figure 2.

Users must make an explicit subjective evaluation of the resources on the web page in order to score their preferences for resources. Implicit behavior, on the other hand, does not require users to make subjective judgments, and some website actions are recorded. We can combine display tracking with implicit tracking to better grasp the user's interest, using display tracking to obtain the static user's interest and implicit tracking to obtain the dynamic user's interest. The collaborative filtering recommendation algorithm makes recommendations to target users based on their closest neighbors' preferences. When determining the target users' nearest neighbors, it calculates the similarity between the target users and other users in the user group and then chooses the *K* users with the greatest similarity to form the target users' nearest neighbors. The collaborative filtering recommendation algorithm is based on the assumption that people have similar behaviors and will make similar decisions. The user's choice contains information about the user's interests. The algorithm calculates the similarity between users by analysing which items' users evaluate, generate the user set with the most similar interest to the current users, predict the current users' rating on the items by using the item ratings in this user set, and finally obtain the recommendation list and make recommendations. When CF recommends users, the main process is divided into three parts: constructing a scoring matrix, finding the nearest neighbors, and generating recommendations.

### 3.3. CF-Based Recommendation System for English Instructional Resources Management

The overall goal of the English instructional resource management recommendation system in this study is to realize the digital instructional resources that can be used by teachers and students in multicampus conveniently under the environment that conforms to the overall planning and design of the construction unit. The core of personalized network instructional resource system is recommendation module, which determines the performance of personalized network instructional resource system to a great extent. The key of recommendation module is to choose an appropriate personalized recommendation algorithm, which can effectively integrate with application fields, reduce possible problems, improve recommendation quality, and reduce the complexity of the system. The traditional recommendation of instructional resources focuses on the main body, while ignoring the interrelation between instructional resources. Aiming at the problems existing in CF and instructional resource recommendation, this study comprehensively considers the relationship between resources and the characteristic behavior information of users themselves to improve the algorithm. First, the learner's behavior and information are digitally modeled to form a model. Then, according to the current system situation, the filter strategy is selected, and the learner's behavior influencing factors are added to form the nearest neighbor set. Finally, online recommendation of learners in various media will be conducted, and the interaction between learners and the system will have an impact on the whole recommendation system, thus forming an organic whole repeatedly. In order to solve the cold start problem in recommendation system, that is, how new users recommend personalized resources to users without any interest preferences and associated friends, this study adopts content-based recommendation algorithm to solve this problem. In a recommendation system based on collaborative filtering technology, the input data can usually be expressed as a user-item evaluation matrix *R* with *m∗n*, as follows:

(1) $$\begin{array}{c} R\left(m,n\right)=\left[\begin{array}{cccc} R_{1,1} & R_{1,2} & \ldots & R_{1,n}\\ R_{2,1} & R_{2,2} & \ldots & R_{2,n}\\ R_{3,1} & R_{3,2} & \ldots & R_{3,n}\\ R_{m,1} & R_{m,2} & \ldots & R_{m,n} \end{array}\right]. \end{array}$$

Among them, the rows represent users, with a total of *m* and the columns represent items, with a total of *n*. The value of *R*_*ij*_ represents the evaluation value of the item *j* by the user *i*, which is generally obtained by the user displaying the submission interest evaluation level. For two users *i* and *j*, the resource sets scored by the two users are as follows:

(2) $$\begin{array}{c} I_{u}=\left\{i_{c}|i_{c}\in I\wedge r_{uc}\neq 0\right\},\\ I_{v}=\left\{i_{c}|i_{c}\in I\wedge r_{vc}\neq 0\right\}. \end{array}$$

The weight function can be expressed as follows:

(3) $$\begin{array}{c} f\left(u,v\right)=\frac{{\left|I_{u}\cap I_{v}\right|}^{2}}{\left|I_{u}\right|\times \left|I_{v}\right|}. \end{array}$$

At the same time, the Pearson correlation coefficient modified by the weight function is shown in the following formula:

(4) $$\begin{array}{c} {\text{Sim}}_{p}\left(u,v\right)=\frac{{\left|I_{u}\cap I_{v}\right|}^{2}}{\left|I_{u}\right|\times \left|I_{v}\right|}\frac{\sum_{i\in I_{UV}}\left(R_{ui}-{\bar{R}}_{u}\right)\left(R_{vi}-{\bar{R}}_{v}\right)}{\sqrt{\sum_{i\in I_{UV}}{\left(R_{ui}-{\bar{R}}_{u}\right)}^{2}}\sqrt{\sum_{i\in I_{UV}}{\left(R_{vi}-{\bar{R}}_{v}\right)}^{2}}}. \end{array}$$

In the calculation of similarity, users' preferences for user resources can be used as a vector to calculate the similarity between users. The similarity is judged according to the distance between two vectors. The smaller the distance, the greater the similarity between them. Traditional CFs generally only recommend users according to the scoring matrix, but in the instructional resource system, the user scoring data are less than the resource scale, so the overall scoring data are sparse. Aiming at this problem, this study considers the attribute characteristics of resources. When a user generally gives a high rating to the resources with certain attributes, it can be considered that the user prefers such attributes. By comprehensively measuring user similarity through scoring similarity and resource attribute preference similarity, we can mine users' potential points of interest, increase data density, and alleviate data sparsity. By constructing a discipline classification tree as the basic structure of instructional resources classification and user tag data, the system labels users by using the professional direction selection and interest topics when users register or log in for the first time, and the skimming data come from the classification tree. User model updating is to improve the original model according to the explicit or implicit feedback from users. In this way, the model can be well matched with the latest preferences of users, thus improving the accuracy and recommendation quality of the model. The system information database is the data source of the whole digital collaborative system. In this model, we collect and record learners' learning behaviors and mine learners' learning behavior trajectories to establish learners' behavior models.

Items *i* and *j* can be viewed as vectors of two *n* dimensions. The similarity of two items is estimated by calculating the spatial angle of these two vectors. For the scoring matrix of *m∗n*, the similarity calculation formula of item *i* and item *j* is as follows:

(5) $$\begin{array}{c} \text{Sim}\left(i,j\right)=\text{cos}\left(\overset{⟶}{i},\overset{⟶}{j}\right)=\frac{\overset{⟶}{i}\cdot \overset{⟶}{j}}{\left|\overset{⟶}{i}\right|\cdot \left|\overset{⟶}{j}\right|}. \end{array}$$

Among them, · represents the vector inner product. The predicted score of the target user *u* to the item *j* is as follows:

(6) $$\begin{array}{c} P_{u,j}=\frac{\sum_{j=1}^{k}\text{Sim}\left(i,j\right)\times R_{u,j}}{\sum_{j=1}^{k}\text{Sim}\left(i,j\right)}. \end{array}$$

Among them, *k* represents the resource set most similar to item *i* in the nearest neighbor table, and *R*_*u*,*j*_ represents the evaluation that user *u* has made on item *j* and the predicted evaluation value obtained by the content-based algorithm. Mainly combined with cross validation to achieve, the formula is as follows:

(7) $$\begin{array}{c} \text{MAE}=\frac{\sum_{g^{\text{test}}\subset G^{\text{test}}}\left|g^{\text{test}}\left(\text{prediction}\right)-g^{\text{test}}\left(\text{authentic}\right)\right|}{\left|G^{\text{test}}\right|}. \end{array}$$

Among them, *g*^test^(authentic) is the real score, *g*^test^(prediction) is the predicted score, and *G*^test^ is the entire set of user scores to be predicted. The system uses recall and precision to evaluate the performance of its personalized recommendation. The formula is as follows:

(8) $$\begin{array}{c} \text{Recall ratio}=\frac{\text{Recommended number of related resources}}{\text{Total number of related resources}}\times 100\%,\\ \text{Precision ratio}=\frac{\text{Recommended number of related resources}}{\text{Number of recommended resources}}\times 100\%. \end{array}$$

The user-item scoring matrix is used in this study to express users' preferences for items, and it is used to implement collaborative filtering recommendation technology. Its advantage is that it is suitable for the representation and establishment of a specific group user model due to group users' interest bias. All users can benefit from the system's recommendation function, which allows both logged-in and non-logged-in users to recommend personalized results and non-logged-in users to capture their interests based on real-time page operations. Learners will rate their satisfaction with a course after completing it, and the data will be saved in the user evaluation database. The accuracy of collaborative filtering recommendations is affected by the detail of the user evaluation database. Users with similar resources have a high degree of similarity in this study. Users in the system are clustered based on scoring information and resource attribute information, and clustering technology is applied to collaborative filtering recommendation. Users who have similar resource attribute preferences are grouped together. Finding the nearest neighbor in several clusters near the target user reduces the space-time cost of neighbor search, alleviates some scalability and real-time issues, and improves recommendation efficiency and quality. The personalized network instructional resource system actively provides recommendation resources to users based on their registration information and behavior characteristics after the introduction of personalized recommendation technology, transforming users from passive browsers to active learners.

## 4. Result Analysis and Discussion

The comparison experiment of the model and algorithm, as well as the analysis of the results, is the main focus of this chapter. This study designs an evaluation experiment for the model and algorithm to quantitatively obtain the recommendation index of the recommendation model after the English instructional resource management recommendation system has been implemented. This will allow us to gain a better understanding of the recommendation model's benefits and drawbacks, as well as serve as a guide for optimising the model's parameters and further optimisation. The system has 100 users registered, and a database of 100 users' personality traits has been created. The instructional resource database has a scale of 200 and 50 interest groups. The top ten English instructional resources with the most similarity are chosen and made available to the appropriate users. The experiment data come from the user operation log in this system, which is used to train the homepage recommendation module. The system will call each module to calculate the recommendation degree of this instructional resource to the user and then save the recommendation degree and the user scoring characteristic value into the database, when the user browses the detailed page of instructional resources and scores the instructional resources.  Table 1 lists the experimental setup.

The function of the instructional resource retrieval module is to receive users' retrieval requests. First, users express their query requirements as keywords or search expressions and input them into the system through the user interface. After the system receives the user's search words or search expressions, the traditional database management system will find out all qualified instructional resources from the instructional resource database according to the matching of the query fields, and form the search results. In the experiment, the sparse level of the data set is also considered, which is defined as the percentage of items in the user-item scoring matrix that are not scored.  Figure 3 shows the subjective rating results of users on recommended resources of different recommendation systems.

It can be seen that the recommended results of English learning resources in this system are more in line with users' needs and preferences, so its score is higher. In addition, the evaluation algorithm, as a standard to measure the recommendation effect of recommendation system, plays a very important role. Therefore, the selection of evaluation algorithms and the characteristics of different evaluation algorithms need to be taken into account, so as to comprehensively evaluate the recommendation effect of a recommendation system. At the same time, it can compare with other recommendation systems comprehensively and get a comprehensive understanding of the recommendation effect of the recommendation system.  Figure 4 shows the comparison of different algorithms when selecting different sparsity.

As can be seen from Figure 4, the improved CF is more accurate than other algorithms because it adds the user behavior weight calculation when the sparsity is small. In this experiment, the average absolute error and recall rate, which are the most widely used and intuitive statistical accuracy measurement methods, are used as evaluation criteria. During the experiment, the data set is divided into a training set and testing set. The algorithm works in the training set and predicts the items in the testing set through the data in the training set. The comparison algorithm used in this study is the classic user CF and project CF. The average absolute error results of different algorithms are shown in Figure 5. The recall results of different algorithms are shown in Figure 6.

The smaller the absolute error value, the higher the recommendation quality. The higher the recall rate of the algorithm, the better the performance of the algorithm. From the comparison results of the average absolute error and recall rate of the evaluation algorithm, it shows that the recommendation algorithm in this study is more accurate than the project CF and the user CF in recommending instructional resources.  Table 2 lists the experimental results of filtering evaluation indexes.

Using the collected data set, under the condition of the same training set and testing set, the recommendation accuracy of different models is compared, and the nearest neighbor size is adjusted to make it produce the best effect in the recommendation process as much as possible. The recommended accuracy results of different models are shown in Figure 7.

The results show that the recommendation accuracy of this model is high. The average filtering accuracy of this system is slightly higher than that of the control experimental system. The main reason is that the former filters instructional resources according to the personalized characteristics of users, and the results are more targeted. Therefore, the model designed in this study, which has the learning function of users' personality characteristics and comprehensive filtering function, can effectively improve the recall and precision of personalized retrieval and personalized recommendation in English instructional resource service. Through the analysis of various experimental data, it can be seen that the English instructional resource management recommendation system constructed in this study is stable. The algorithm's recall rate can reach 96.37%, and the recommendation accuracy rate is as high as 95.31%, which is higher than the traditional method's 6.37%. The English instructional resource management recommendation system constructed in this study has good performance in all aspects and effectively improves the satisfaction of resource users. It can effectively provide high-quality resources for English teaching and can better satisfy users' experiences.

## 5. Conclusions

This study examines the use of personalized recommendation systems and digital English instructional resources, as well as the principle, recommendation process, and classification of collaborative filtering recommendation algorithms. This study has conducted extensive research on the topics of sparsity, cold start, and scalability of collaborative filtering recommendation algorithms, as well as proposed solutions. A CF-based English instructional resource management recommendation system is designed and implemented as a result of this. This study describes in detail the key technologies used in the system, presents the overall framework and functions of the digital English instructional resource system, and designs and implements a personalized recommendation module in the instructional resource system based on the learning habits and instructional resources of users. The system's advancement allows for better sharing and reuse of digital resources, as well as the discovery of instructional resources that learners may be interested in. The system's usability, ease of use, stability, and high real-time performance are demonstrated through the running test and performance analysis, and the system's convenient capacity expansion for many times in the future is also demonstrated. According to the research, this algorithm has a recall rate of 96.37% and a recommendation accuracy rate of 95.31%, which is higher than the traditional method's 6.37%. The English instructional resource management recommendation system developed in this study performs well in all areas and effectively increases resource users' satisfaction. It has the potential to effectively provide high-quality resources for English teaching while also improving user satisfaction. However, because the digital English instructional resource system is a complex learning platform with time and technology constraints, there are still some issues in the system's research and development that need to be addressed. The balance between the real-time performance of the recommendation system and recommendation quality is the focus of the following work. Additional research into the characteristics of educational resources is necessary to expand the user interest model and instructional resource model.

## Figures and Tables

**Figure 1:** Digital college English instructional resource management model.

**Figure 2:** Improved structure of English instructional resource management recommendation system based on CF.

**Figure 3:** Comparison of users' subjective ratings.

**Figure 4:** Comparison of algorithm results when selecting different sparsity.

**Figure 5:** Average absolute error results of different algorithms.

**Figure 6:** The recall results of different algorithms.

**Figure 7:** Recommended accuracy results of different models.

**Table 1:** Experimental environment settings.

Category	Setup
Processor	Dikaryon
Internal storage	512
Hard disc	80 GB
Operating system	Windows
Development platform	MyEclipse
Program	Java
Database system	MySQL

**Table 2:** Experimental results of evaluation index.

Model	Average precision rate (%)	Average recall rate (%)
Weighted association rule recommendation model	89.34	91.42
User-based recommendation model	84.12	86.37
Content-based recommendation model	82.36	85.24
Recommended model proposed in this study	95.36	96.17

## Data Availability

The data used to support the findings of this study are available from the corresponding author upon request.
